# Structural Modifications and Strategies for Native Starch for Applications in Advanced Drug Delivery

This article has been retracted.

**DOI:** 10.1155/2022/2188940

**Published:** 2022-08-10

**Authors:** Pankaj Bhatt, Vipin Kumar, Richa Goel, Somesh Kumar Sharma, Shikha Kaushik, Shivani Sharma, Alankar Shrivastava, Mulugeta Tesema

**Affiliations:** ^1^KIET Group of Institutions (KIET School of Pharmacy), Delhi NCR, Muradnagar, Ghaziabad, India; ^2^Department of Pharmaceutical Science, Gurukul Kangri (Deemed to Be University), Haridwar, Uttarakhand, India; ^3^Department of Pharmaceutics, KIET Group of Institutions (KIET School of Pharmacy), Delhi NCR, Muradnagar, Ghaziabad, India; ^4^School of Pharmacy and Research, Dev Bhoomi Uttarakhand University, Dehradun, Uttarakhand, India; ^5^Department of Chemistry (Analytical), College of Natural and Computational Sciences, Dambi Dollo University, Dambi Dollo, Oromia Region, Ethiopia

## Abstract

Pharmaceutical excipients are compounds or substances other than API which are added to a dosage form, these excipients basically act as carriers, binders, bulk forming agents, colorants, and flavouring agents, and few excipients are even used to enhance the activity of active pharmaceutical ingredient (API) and various more properties. However, despite of these properties, there are problems with the synthetic excipients such as the possibility of causing toxicity, inflammation, autoimmune responses, lack of intrinsic bioactivity and biocompatibility, expensive procedures for synthesis, and water solubility. However, starch as an excipient can overcome all these problems in one go. It is inexpensive, there is no toxicity or immune response, and it is biocompatible in nature. It is very less used as an excipient because of its high digestibility and swelling index, high glycemic index, paste clarity, film-forming property, crystalline properties, etc. All these properties of starch can be altered by a few modification processes such as physical modification, genetic modification, and chemical modification, which can be used to reduce its digestibility and glycemic index of starch, improve its film-forming properties, and increase its paste clarity. Changes in some of the molecular bonds which improve its properties such as binding, crystalline structure, and retrogradation make starch perfect to be used as a pharmaceutical excipient. This research work provides the structural modifications of native starch which can be applicable in advanced drug delivery. The major contributions of the paper are advances in the modification of native starch molecules such as physically, chemically, enzymatically, and genetically traditional crop modification to yield a novel molecule with significant potential for use in the pharmaceutical industry for targeted drug delivery systems.

## 1. Introduction

Starch has been utilised in everyday life for centuries. Egyptians generally used cooked flour of various cereal pastes which was diluted with vinegar to prepare cement papyrus strips, although the early Chinese public covered the papers with starch which had less viscosity when gelatinized to avoid ink permeation. Carbohydrate chemists began synthesising several starch compounds in the 1930s, considerably expanding starch's utility. Starches are essential carbohydrates which are included in our nutritional intake and come from a variety of environmental sources which can be listed as such as rice, wheat, potato, maize and wheat, potato, rice, maize, and tropical plants. They have a wide variety of qualities that help to obtain the preferred quality of food products. Due to the limitations of raw starch obtained directly from natural sources, during processing, some of its characteristics being resistance to high temperature, viscosity, and thermal disintegration, the food industries have a preference for starches with superior behavioural qualities [1].

Starches are carbohydrates composed of primarily of two components called amylopectin and amylose. This biodegradable and nontoxic biopolymer is abundant in nature and creates consistent pastes and gels when heated in the presence of adequate water. As a result, starch is widely considered as an industrial ingredient in large quantities in a wide range of industries including chemicals, petrochemicals, pharmaceuticals, bioethanol, food, feed, paper, cloth, laundry finishing, construction resources, and other decomposable products [2].

Free fatty acids and lipids present in the form of phospholipids in starch [3] and tend to form complexes with amylose and amylopectin and form starch granules with less solubility [4]. Their end products are opaque and low-viscosity pastes [5] which significantly reduces the property of the starch particles [6]. Hence, starch is considered as biocompatible and nontoxic, although LC50 is characterised as toxic when 50% embryos die at a conc. of 1 mg/ml equal to 1000 mg/l [7]. Excipients have traditionally been thought of as inactive chemicals that serve as binders, sweeteners, disintegrants, and adhesives in oral delivery systems [8].

In the past decades, to enhance patient amenability, biocompatibility, and effectiveness, more importance has been given to the effects of excipients on formulation and to the decrease in the use of synthetic/chemical grade excipients in pharmaceutical formulations [9].

Excipients have been proven in studies to change the rate at which the drugs are released from the formulations, hence changing the system's efficiency and the active pharmaceutical ingredients absorption. As a result, there is a growing trend in the direction of use of naturally obtained excipients, sometimes known as “herbal excipients” [10]. The extracts of the plant and their useful properties may prove helpful in pharmacological studies possessing large amounts of bioactive constituents, which can be used for the preparation of therapeutic and health promoting formulations which may provide future drugs for dreadful diseases [11]. Being biologically active, phytochemical constituents are natural compounds found in plants which protect them from diseases and damage [12].

Inappropriately, starches have limited functionality in their natural state, which can make them difficult to use. The temperature of gelatinization, digestibility, rheological properties, crystalline quality, different amounts of water absorbed at different temperatures, pasting capability, and strength of the gel are only a few of the properties that each starch source has. Due to the paucity of economical sources, modified starches have been frequently prepared and used to improve quality and overcome various limitations of native starches, henceforth broadening their use in industry. Modification methods can alter a variety of features including gelatinization, swelling, solubility, pasting and retrogradation quality, digestibility, and rheological properties, among others [13]. As a result, many forms of starch alterations are used to enhance the structural, physical, and functional qualities for precise utilisation of starches.

Chemical alteration procedures are most commonly carried out in industry because they are efficient in cost and simple to use. The three accessible -OH functional groups (at C2, C3, and C6 positions) (at positions C2, C3, and C6) [14] of the molecular structure can be transformed with a few chemical modifications named etherification, esterification, and/or oxidation in the most widely used chemical procedures [15]. The amount of alteration in each of the three groups varies based on the genetic origin and synthesis conditions [16]. By modification of starch, gelatinization, swelling, solubility, pasting, and retrogradation are the few properties which are affected [13]. Compared to its natural form, these newly developed features allow the altered starch to be considered for use for pharmaceutical purposes, such as the use of it as an excipient. Demat form and screened starch is frequently used as a stabilizer in the wet gelation process, and it is an important component in the formation of capsules, tablets, and other dry dosing schedules [17]. A disintegrant is a pharmaceutical excipient used to break down solid dose forms such as granules, tablets, or into smaller discrete particles. The origin or type of starch determines the degree of swelling, which is symptomatic of the relative contribution and structure of amylose and amylopectin in the particular starch [18, 19].

The weak associated interactions of starch can indicate its disintegrating ability [20], which is caused by the creation of holes via which liquids can permeate the dry active ingredient, enabling the medicine to dissolve. Starch absorbs moisture between 10 and 17 percent when acclimatised to typical ambient air due to its hygroscopic characteristics [21].

As a result, this paper examines the different processes to alter the various properties of the native starch. From the plant sources, native starch with minimal treatment was obtained [22]. Starch is constant in storage for longer periods [23]. Native as well as modified starches are used as pharmaceutical excipients because of their soft dryness, gelling, and viscosity providing properties [17].

## 2. Physical Modification

In the food industries, physical changes are applied since they do not require any chemical entity for reaction processes. Several new technologies have emerged in the physical modification of starch. Deep freezing, osmotic pressure treatment, and dry heating are few of the latest physical alterations that have been researched in the recent decade [24]. It does not cause the D-glucopyranosyl units of the starch molecules to be modified. Physical modifications simply modify the structural arrangement of starch molecules inside the granules and the complete arrangement of the granules. These alterations in granules have an impact on starch characteristics such as paste and gel properties and even digestibility [25] as presented in Table 1.

Miller and Huber [24] studied the results of three different studies and reported changes in the properties of starch which are affected by osmotic pressure treatment. These changes were due to the heating of the starch in an osmotrophic solution which reduces granule gelatinization and swelling; hence, osmotic pressure treatment is a type of hydrothermal treatment. Szymonska and Krok [26] and Szymonska and Wodnicka [27] reported that recurrent thawing and freezing of potato starch granules of 13% moisture resulted in surface erosion, increased surface area, mean pole diameter, and total micro- and mesovolume. Chiu et al. [28] heated starch with <15% moisture at a temperature of 100C and the temperature at which thermal degradation occurred, and it formed products with shear, acid, and temperature tolerances related to those of chemically cross-linked starches. The transformation was due to low moisture content and alkalinity. Fluidized bed is a way to heat starch, but this process has only been investigated with amaranth [29].

The changes in the molecular structure of starch samples have been studied through FT-IR, and X-ray diffraction results are shown in Figures 1 and 2. The results inferred that the molecular structure of the starch is being changed and due to that the various properties of the native starch are also altered [27].

Pukkahuta et al. studied through SEM results (Figure 3) that there is no variance between native and heat moisture treated potato starch, but osmotic pressure-treated potato starch causes changes in the granular morphology of the pretentious granules, and these seem to have folded structures with their outermost side down inwards, looking like donut's shape. This transformed morphology of granules are because of the effect of osmotic pressure treatment is called “plasmolysis” [31].

## 3. Enzymatic Modification

Hydrolysing enzymes have been widely used in enzymatic modifications [25]. The distribution of branch chain length, molecular mass of amylose/amylopectin, and percentage of amylose/amylopectin are the properties that are altered by the enzymatic modifications of natural starch. Designing a starch with a specific and unique structure of starch can be processed by enzymatic reactions which occur when the gelatinized starch reacts with the provided enzyme to form upgraded starch. For enzymatic starch alterations, it is one of the modification procedures as discussed in Table 2. For a variety of food and nonfood uses, these processes usually result in starch with modified physicochemical properties and structural qualities [35]. The less well-ordered amorphous sections in the structure are more vulnerable to enzymatic replacement, but the most resistant part to enzymatic treatment is crystalline lamellae [36, 37].

Hydrolytic enzymes, also known as hydrolases, break different groups of biomolecules such as esters, glycosides, and peptides. They break down lipids, nucleic acids, proteins, carbohydrate, and fat molecules into their simplest units [38]. The proportion of different components of enzyme and the source of the enzyme influence the rate of enzymatic [39]. Lignocellulose enzymatic hydrolysis has long been studied as a method to depolymerize the biomass into fermentable sugars and conversion to biofuels and biochemicals [40] Cellulose to glucose enzymatic hydrolysis has received increased interest over the last 10 years. The growing demand for economically sustainable biofuels specifies an urgent need for reducing the costs related to their production [35].

As per Li et al., native rice starch grains are polyhedral, angular, and irregular, and the surfaces are smooth with no cracks as displayed in Figure 4. Due to gelatinization and retrogradation of the modified starches, the granular structures get disappeared completely. A-MS has continuous irregular spongy structures with continuous network. These have pores and loose structure, but the structures of A/PUL-MS have fewer holes and small pore size and have dense layered structure compared to the A-MS, whereas A/STE-MS has no surface holes, and the granular structure is very dense which appears like a stone [42].

Jiang et al. have found the alteration in the rheological properties of normal starch and enzymatically modified starch as shown in Figure 5. The unmodified starches have the greater viscosity compared to the modified one, and the viscosity of starch keeps on decreasing with the increase in the reaction time with 4*α*GT [41].

## 4. Genetic/Biotechnological Modification

The alteration in genetic material of the plant or biotechnological alteration of plant DNA is referred to as genetic modifications. The enzymes responsible for the production of starch are targeted by transgenic technology; thus, it is considered a genetic alteration technique which can also be done through traditional plant breeding techniques or biotechnology [46]. Plant biotechnology breakthroughs have created a good prospect to increase the quality of starch in various crops. Starch is not only a common dietary carbohydrate [47] but also a low-cost, renewable raw resource utilised to make varieties of vital products, e.g., paper, textiles, medications, construction materials, and nutraceuticals [48]. Multiple aspects of starch can be changed through genetic manipulation, including morphological characteristics, crystallinity, gelation temperature, amylopectin and amylose ratio, and the number of phospholipids. In general, there are three types of genetic alteration of crops that can be done, e.g., traditional crop modification, genetic engineering, and genome editing [49].

Plants generate a range of proteins, including mammalian antibodies, blood substitutes, vaccines, and some other therapeutic substances using gene editing, which has led to a renaissance of interest in getting novel pharmaceutical molecules from botanical extracts [23]. Foreign protein production from genetically engineered plants has recently emerged as a viable alternative to microbial fermentation or mammalian cell culture. Plants genetically engineered to function as bioreactors can create fusion proteins in larger numbers than mammalian cell systems [50]. Traditional therapeutic immunotherapies were produced in rodents by the body's immune system; however, these molecules were quickly detected as foreign, restricting the value of such inhibitors for therapeutic usage, especially with chronic exposure. Aside from the absence of anaphylaxis or serum sickness, the presence of neutralising antibodies that inactivate the medicine frequently precludes future therapeutic usage. While innovative technologies have enabled the replacement of murine antigens with substantially humanised or chimeric antigens and the synthesis of full human antigens [42], polio vaccines, like conventional food vaccines, employ whole, weakened microorganisms or semipurified substances to promote both systemic (Ig-G) and local membrane (Ig-A) protection. Plant vaccines may produce complete proteins, but the use of DNA encoding just specific antigenic regions from bacteria, harmful viruses, and parasites has garnered a lot of interest [51].

## 5. Traditional Crop Modification

The traditional methods of modification of the plant such as selective breeding and cross-breeding are one of the processes in which plant breeding is used to selectively develop a particular phenotypic trait by selecting which male and females will reproduce and have offspring together.

### 5.1. Genetic Engineering

It is basically a method in which authorized experts copy a particular gene with a look for a trait from one plant and put it into the other plant in which the desired characteristics are incorporated, and it builds the scientific advantages through DNA technology.

### 5.2. Genome Edition

Genome edition is a novel approach that allows some researchers to generate new crop types in a more precise and targeted manner. The use of a genome editing tool makes modifications easy and efficient that were previously possible through traditional breeding [52].

## 6. Chemical Modification

It is done by attaching a functional group in to the molecular structure of starch in its natural state resulting in specific physicochemical properties for the starch molecule. These alterations influence the retro gradation, pasting ability, proximal composition, and gelatinization of unmodified starch granules [53]. At various sites and locations of unmodified starch, the stability of intra- and intermolecular interactions are increased due to these alterations which are carried out with the help of various chemicals. The other chemical and functional properties of altered starches are affected by the amount of starch supply, degree of substitution, synthesis environment, types of starch used, and the circulation of their placing agents throughout the starch molecule. The derivatization methods that are used for chemical alterations are oxidation, acetylation, cross-linking, acid hydrolysis, cationization, etc. [54].

The starch is recyclable and the existence of particular functional groups and the macroscopic structure of starch are all factors that influence its sensitivity towards modification. Furthermore, regarding chemical modifications subjected to the position of -OH group and alpha-1, 4-glycosidic bonds versus alpha-1,4-glycosidic bonds and alpha-1,6-glycosidic bonds in starch have different properties. Primary alcohols have a hydroxyl group at carbon C6, whereas secondary alcohols have a hydroxyl group at carbons C2 and C3. Unmodified starch is a triol compound which can be converted to hemiacetal whenever the glucose ring component –CHOH–CHOH– replaces the carbon atoms at C2 and C3 positions. The existence of three -OH groups in glucose renders it amenable to replacement processes allowing for a wide range of starch alterations. The reactivity of starch is also affected by its grain size. The susceptibility to modification increases with the size of the grains. This is due to the fact that external influences have comparatively easier contact with larger grains. Modification is the procedure of altering normal properties through physical, chemical, or enzymatic processes [55].

## 7. Oxidation of Starch

The most commonly used alteration technique to obtain specific changes in molecular structure is the oxidation of starch. In this process, the primary and secondary –OH groups present in the glucose molecule led to the development of aldehyde or carboxyl groups. The efficiency of the oxidation reaction is determined by the nature of the oxidant, the biological origin of the starch, and the procedural parameters. Furthermore, the oxidation method can affect the intermolecular bonds and/or fractional depolymerisation of polymer chains present in the starch molecule [55]. Typically, the properties of starch are altered by carrying out a reaction of the slurry of starch with an oxidising agent at a particular temperature and specified pH [56]. The three most accessible -OH groups react with the oxidising agents throughout the oxidative process to create new starch derivatives. The oxidative technique and reagents are considered a parameter to govern the type and quality of the oxidised starch derivative. As a result, the native starch-derived physicochemical properties are improved [57].  Table 3 shows the oxidation of starch and the change in its properties after modification. Oxidised starches are widely used in the paper industry to improve paper strength and processability. It is also used in the finishing, textile, laundry, construction materials, and culinary sectors. The major purpose of oxidised starch seems to be in the pulp and leather sectors; nevertheless, due to its low viscosity and high stability, clarity, film forming, and bonding quality, which have been employed in food coatings, its usage inside the food sector is expanding. The oxidation approach for starch alteration is an essential procedure in which absorption bands such as carbonyl and carboxyl groups are inserted into the starch granules for depolymerization [54] despite the fact that proper conditions, such as temperature and pH, must be maintained during oxidation. The aggressive oxidants utilised are hydrogen peroxide, peracetic acid, potassium permanganate, sodium hypochlorite, chromic acid, and nitrogen dioxide [55, 56].

In recent years, oxidised starch has been widely used in the food sector to create adherent surfaces and coatings [57]. Because of partial macromolecule decomposition in oxidised starches, they have reduced hot paste viscosity, a lesser susceptibility to syneresis due to bulk carbonyl and carboxyl groups, whiter granules, and more translucent pastes [58]. Reagents that generate ether or ester linkages with hydrophilic groups in starch granules play an essential role in bridge starch [59]. This alteration increases the stiffness of the polymer by producing a three-dimensional web. Cross-linking increases the degree of polymerization and molecular mass in starch. Aside from the origin of the starch molecules, the methods and settings utilised for covalent modification have a considerable influence on the end product's quality. Cross-linking affects the paste clarity and swelling capacity [60, 61], because of the pastes' stabilising, hardening, purity, and thermal decomposition qualities. Crucifix starch is related to frozen pharmaceutical preparations in the food business, as well as being employed in other sectors such as polymers [62].

As reported by Lima et al.  Figure 6 represents the amylose content in native and oxidised starch, and it gets reduced with the increase in the reduced sugar, and the amount of amylose present in the modified starch also depends on how long the starch is being treated with ozone [66] .

According to Barbosa et al., there are structural changes in potato starch as presented in Figure 7 which are due to the reduction in the basic viscosity of the starch as the amount of H_2_O_2_ is increased, and it is significant if the molecular weight is reduced. It occurs due to breakage of glycosidic bonds during the reaction and consequently, due to modification. However, the oxidation reaction is not at all easy to identify due to bands' overlapping and suppression. Therefore, a 2nd derivative process is carried out on the spectra to develop the sensitivity for the possible changes in chemical structures which are changed during process. In Figure 8, the 2nd derivative values of band behaviour as a function of oxidant concentration have been shown for the wavenumbers 2930, 2887,1460, 1244, and 1144 cm^−1^ [53].

## 8. Esterification of Starch

It is a procedure in which three easily accessible -OH groups of starch molecules are converted to alkyl or aryl derivatives. This alteration process usually affects various properties, and one of the most important is its retro gradation ability resulting in reduced in-between amylase connections with the outside chain of amylopectin [68]. This category includes a number of techniques and acetylation in one of the techniques which is most frequently used. This technique is extensively employed in the biotechnology, food industry, and fabric sectors [69]. On the basis of the degree of substitution, acetylated starches are characterised into three different forms (DS), which are listed as low DS, medium DS, and high DS starches. Small degrees of substitution starch by acetyl group are the most prevalent type of acetylated modified starches. These low DS starches have a degree of substitution value of 0.01% to 0.2% and are cold water soluble [70]. Starches in medium DS are usually water-soluble at room temperature but not as much as low DS starches and have a degree of substitution of 0.3% to 1%. The solubility of high degree of substitution acetylated starches is not well in water but have a very good solubility in organic solvent, and the degree of substitution is 2% to 3%. The effectiveness and amount of acetylation are determined by the starch type's ultrastructure, which varies based on the botanical origin, as well as the reaction conditions. The changed properties after esterification of starch are shown in Table 4 [4].  Figure 9 shows the FT-IR spectra of citric acid and native starch FT-IR-treated starch.

Wu et al. reported that citrate-modified raw starch of canna is different from the citrate modified starch, because a new peak is observed by them in the modified starches at 1740 cm^−1^. This new absorption band is linked to the extending vibration of C=O bond of the carboxylic acid group. With the increase in the degree of substitution of citric acid, the peak at 1740 cm^−1^ becomes stronger. These results confirm the esterification reaction carried out between canna, starch molecules, and citric acid [75].

Lee and Chang reported that the shapes of maca starch granules as shown in Figure 10 are oval or round with being smooth in shape and are consistent with the previous studies. However, esterified maca starch with citric acid shows some of the irregular surfaces and some wrinkles and dents with irregular oval and doughnut shapes. They reported that the morphological properties of the esterified granules were almost the same in accordance to previous study [71].

## 9. Conclusion

However, these physical and chemical alterations may limit starch's utility in some formulations while enhancing its functional quality in others. Functionalizing delivery systems with these physicochemical features create new possibilities for enhancing the overall efficacy of starch related systems. The most common starch modification methods are chemical modification methods, which basically include esterification and oxidation and few other modification techniques. These are the modification methods which can alter various properties of starch like digestibility, chemical bonds, molecular structure, amylose, and amylopectin chain, and these can be altered according to the necessity of the properties which are required. In essence, physical modification shows that it significantly alters the physical properties of starch such as the morphology of granules or viscosity of the starch paste. Altering these properties can be beneficial for a targeted drug delivery systems. Genetic and enzymatic are other techniques which are also capable of altering the various properties of starch enzymatic modification and are also used to alter the nutritional content or gelatinization properties or granule morphology. Although enzymatic modifications which alter the properties in a similar fashion as chemical modifications but carrying out an enzymatic reaction is not feasible and cannot be performed without professionals, chemical modifications are preferred over enzymatic modifications. The genetic modification alters with the plant genetic material and the properties of starch automatically get modified in its native form itself. Furthermore, this modified starch can be used in the formulation of novel drug delivery systems or in the preparation of various products according to the needs. If the chemical modifications were enhanced, novel drugs were isolated in the future having potential for use in the medical industry for a targeted drug delivery system.

## Figures and Tables

**Figure 1:** Models of X-ray diffraction of different starch samples: (a) frozen oven-dried. (b) Oven-dried and frozen without the use of water. (c) The ratio of water to oven-dried and frozen is 1 : 1.5 and 1 : 1. (d) Oven-dried and mixed only with water, but not frozen. (e) Dried and not frozen in the air. (f) Dried and frozen in the air [27].

**Figure 2:** FT-IR absorption spectra of potato starch: (a) oven-dried and iced up with water in the ratio of 1 : 1.5; (b) oven-dried and not iced up [27].

**Figure 3:** SEM of starch granules of potato. (a) Potato native starch. (b) Moisture heat treatment of starch sample (120°C, 60 min). (c) Osmotic pressure treatment with potato starch (120°C, 60 min) [31].

**Figure 4:** SEM results of (a) native rice starch (NRS), (b) autoclaved developed starch (A-MS), (c) autoclaved/pullulanase–changed starch (A/PUL-MS), and (d) autoclaved/sequential three enzymatic–modified starch (A/STE-MS) [42].

**Figure 5:** Viscosity of 4*α*GT-treated starch with different concentrations of 4*α*GT [41].

**Figure 6:** Apparent amylose and reducing sugar contents [66].

**Figure 7:** FT-IR of native and oxidised (H_2_O_2_ treated) potato starch [53].

**Figure 8:** 2nd derivative FT-IR band behaviour as a function of the oxidant concentration [53].

**Figure 9:** FT-IR spectra of native- as well as citric acid-treated starch [9].

**Figure 10:** SEM of and esterified and native maca starch with citric acid [71].

**Table 1:** Different physical modifications and properties changed after native starch modification.

Starch type	Technique(s)	Modification method	Properties changed	Reference
Rice starch	Heat and moisture treatment	It is performed at the moisture content of 25%, then allowed to stand at 4°C for 24 hrs, transferred to screw stainless steel nonstop, then heated with oil for 4 h at 110°C, and then dried at 40°C.	Digestibility, physiological index, nutritional content, biochemical indices	[30]

Potato starch	Osmotic-pressure treatment (OMT)	100 g of dry starch is suspended in Na_2_SO_4_ solution, kept in the autoclave at 105°C and 120°C at 328 and 341 bar, respectively, kept for a particular period of time, and then cooled to room temperature; excess chemicals are removed by rinsing through distilled water, finally centrifuged, and then dried at 40°C.	Microscopy, thermal properties, particle size, pasting properties, viscosity, water holding strength,	[31]

Potato starch	Deep freezing	Starch which is dried through an oven is immersed in liquid N_2_ kept in an open container for a particular period of time, then the nitrogen is allowed to evaporate, and the sample is allowed to warm up to the room temperature for a while.	Molecular structure, chemical composition, thermal properties, diffraction patterns, viscosity	[27]

Corn starch	Pulsed electric fields treatment	Deionized water is added to the suspension of native corn starch (8% *w*/*w*) along with KCl to maintain a 200 *μ*S/cm electric conductivity. The sample is then exposed to different levels of PEF where it is filtered and dried at 40°C afterwards.	Particle size distribution, diffraction pattern, viscosity, granulation, size, denaturation, and molecular rearrangement	[32]

Waxy maize and potato starch	Thermally inhibited treatment (dry heating)	Firstly, starch is partially hydroxypropylated; then xanthan gum was added to water with constant stirring. The prepared gum solution is added to the starch, mechanically stirred for a specific period, and then dried in a hot air oven to maintain a moisture of <10%; then the mixture of starch and gum is heated at 130°C for 2-4 h.	Viscosity, pH of the mixture, pasting properties, light transmittance, paste clarity	[33]

Maize starch	Superheated starch	A mixture of demineralized water and starch in 5 : 1 is heated at the desired temperature in DSC with the rate of increase in temperature to be 10°C/min and cooled rapidly at a rate of decrease in temperature to be 200°C/min to 25°C	Physical characteristics, molecular characteristics, thermal properties, gelling properties,	[34]

**Table 2:** Enzymatic modifications and properties changed after native starch modification.

Starch type	Reagent used	Modification method	Properties changed	Reference
Corn starch	4-*α*-Glucotransferase	Cornstarch is prepared with pH 7.5, 50 mM Tris-HCl buffer solution (8% *w*/*v*), then heated in a water bath at 95°C for a particular period of time, and then the reagent is mixed to the mixture. It is incubated for different time intervals, then immediately kept in autoclave for 30 min. Then, ethanol is used to precipitate out the reagent, centrifuged, washed with the help of deionized water, and then freeze-dried.	Digestibility, amylose content, iodine binding, chain length distribution, molecular weight, structural properties	[41]

Rice starch	Pullulanase	A 20% suspension of native starch is treated with sodium acetate buffer, and then it is gelatinized in a boiling water bath for 30 min; pullulanase (20 U/g) is added and kept at 60°C for 6 h. After that, the mixture is kept in the boiling water bath for a while to stop the enzymatic reaction, and it is cooled at room temperature. Then, stored at 4°C for 24 h. the precipitate is centrifuged and dried in a blast drying oven.	Chain length distribution, surface holes, physiochemical properties, crystalline structure, swelling index, solubility, thermal properties, digestibility, rheological properties	[42]

Amylose starch	Glycogen branching enzyme in *Streptococcus mutans* (SmGBE)	A starch solution is prepared with 1 N NaOH followed by demineralized water and 200 mM buffer consisting of sodium acetate and the pH is raised to 5.0 using hydrochloric acid and then gelatinized and incubated for 1-24 h at 37°C in 600 l SmGBE, then three volumes of ethanol are added to and kept at 4°C for 1 h. and then ppt. Is centrifuged and washed with ethanol followed by vacuum drying.	Branch chain length, molecular weight, retrograde properties, digestibility	[43]

Maize starch	Maltogenic amylase	Starch sample is dispersed in sodium acetate buffer and then the mixture is heated at 90°C for a particular period of time, cooled to 50°C and hydrolysed by Maltogenic amylase at 50°C for the period of time then kept at 95°C for 15 min to finish the enzymatic reaction.	Molecular weight, chain length thermal properties, swelling index, digestibility, branched density.	[44]

Cassava starch	Fungal lipase	Palmitic acid and starch are taken in equal proportion and dissolved in solution (DMF). 200 mg lipase power is added and incubated in a water bath at 40°C for 4 hours; by adding alcohol the sample is precipitated and then is oven dried.	Thermostability, digestibility, swelling power, viscosity,	[45]

Rice starch	*β*-Amylase	20% suspension is prepared with native starch and sodium acetate buffer and then allowed to be gelatinized on a water boiling bath for almost 30 min. And immediately kept in an autoclave at 121°C for an hour, then incubated with the *β*-amylase at 55°C for 15 minutes. Then kept in a boiling water bath to inactivate the enzyme. Stored at 4°C for 24 hr. and ppt. Were separated through centrifugation and dried through blast drying oven	Crystalline properties, chain length distribution, amylose content, thermal properties, digestibility, solubility, swelling index,	[42]

**Table 3:** Oxidation of starch and properties changed modification.

Starch type	Reagent used	Modification method	Properties changed	Reference
Potato starch	Hydrogen peroxide (30%)	The starch is made with the help of distilled water and maintaining pH to 4 with the help of CH_3_COOH and then added H_2_O_2_ dropwise, left it for 8 h, and dried at 45°C for 48 h in a hot air oven.	Viscosity, C-H bonds, crystalline properties, microstructure	[63]

Cassava starch	Ozonation by industrial oxygen	The starch is dispersed in water in 1 : 10 ratio mixture in a glass reactor; then ozone is produced by using ozone generator unit, ozone is passed through the sample and treated for 15-30 minutes.	Solubility, crystallinity, rigidity, tensile strength, opacity	[64]

Rice starch	13-Hydroperoxyoctad-ecadienoic acid	The 10 mg/ml rice starch mixture were incubated using a particular conc. of 13-HPODE at 25°C for 24 h. Unreacted 13-HPODE is decanted, and modified rice starch is lyophilized in its place.	Solubility, oil holding ability, water holding ability, foaming ability, emulsification, foam stability, activity index, emulsification stability index	[65]

Arracacha starch	Ozonation	The ozone in ozone generator unit by the coronal discharge method passed through the starch solution with water kept in a glass reactor and dried in oven at 35°C	Paste clarity, particle size, viscosity, pasting properties, water solubility and absorption indexes, molecular size, apparent amylose content.	[66]

Potato starch	H_2_O_2_ with electrolytic cell	A 50 g starch and 150 ml of 0.1 mol/l Na_2_SO_4_ were taken in an electrolytic cell with magnetic force stirring and a boiling water bath. H_2_O_2_ is added and the current is allowed to flow for a particular period, temperature reduced to 25°C and filtered through vacuum filtration.	Carboxyl content, thermal stability, crystalline properties, viscosity, and chemical bonds	[67]

**Table 4:** Esterification of starch and properties changed modification.

Starch type	Reagent used	Modification method	Properties changed	Reference
Maca starch	Citric acid	Citric acid and native starch are mixed and kept at room temperature for 16 h and dried in a hot air oven to obtain a moisture level of around 5-10%, afterwards, it is dried at 140°C for 4 h before being cleaned with distilled water multiple times to eliminate untreated citric acid.	Digestibility, microstructure, partial size, zeta potential value, stability	[71]

Waxy maize starch	Octenyl succinic anhydride (OSA)	The starch is suspended in purified water and the pH is brought to 8.5 with the help of NaOH, the required amount of OSA (0.5-3% starch) is added slowly and left for 6 hrs. At room temp. Then, the pH were maintained to 6.5 with HCl, then centrifuged, washed, and oven dried.	Digestibility, molecular structure, nutritional properties, swelling properties, solubility, gelatinization, retrogradation	[72]

Waxy corn starch	Dodecenyl succinic anhydride (DDSA)	An emulsion of DDSA and MES prepared by distilled water, finished dried starch is suspended in water, pH is adjusted to 8.5 with NaOH and the emulsion mentioned above is added, after reaction pH is maintained at 6.5-7 by HCl, the mixture is centrifuged and dried in vacuum oven	Wettability, contact angle, water solubility, chemical bonds	[73]

Waxy maize starch	Citric acid	In a ratio of 5 : 2 w/w, starch and citric acid are dissolved in distilled water, respectively, pH is adjusted to 35 with NaOH and kept at normal temperature for 24 h, then esterified at 130-150°C for 3-5 h. it is washed with ethanol and dried.	Digestibility, gelatinization, particle size, microstructure, chemical bonds, clarity	[74]

Corn starch	Folic acid	Firstly, folate is reacted with N,N'-dicyclohexylcarbodiimide and dimethyl sulfoxide, then addition of starch to the reaction mixture and afterwards reacted in dark conditions for 24 h, then the product is washed with 0.1 N HCl, then the unreacted FA is washed out, the finished substance is lyophilized and powdered.	Mesoscopic structure, crystallinity, molecular packing, digestibility, solubility, wettability	[54]

Canna starch (RS4)	Citric acid	Citric acid is dissolved in water and the pH is adjusted to 3.0 with the help of NaOH, the solution is uniformly sprayed on canna starch and the mix is being packed and vacuum treated. The sample were kept in Petri dish and kept in microwave at 55°C for 4 min for microwave treatment, grind powder and IR treatment at 140°C for 1 h. after that, it is rinsed with purified water and then ethanol and in the end oven dried.	Digestibility, optical activity, pasting properties, thermal properties, particle size, and crystallinity.	[75]

## Data Availability

The data shall be made available on request.
